RETRACTED

# Emotional Expression and Playing Psychology in Accordion Playing under Complex Audio Background Environment

**DOI:** 10.1155/2022/2482899

**Published:** 2022-09-12

**Authors:** Xuwei Wen

**Affiliations:** School of Music, Shanxi Datong University, Datong 037009, China

## Abstract

Accordion performance is an emotional art, and the generation of emotions is inseparable from human psychological activities. It has a great relationship with the performance of music and has a great impact on the performance of the performance. The performance of the accordion is a process of psychological perception, understanding, imagination, experience, and emotion. It not only shows the true creative intention and emotion of the “original work” but also integrates it into the individual characteristics of the individual. In the creation, the true artistic vitality is given to each note, thereby enriching the musical composition, thus showing its unique charm. Therefore, this paper proposes a study on the emotional expression and playing psychology of accordion playing. In the end, the performance of class A students was significantly better than that of class B students, while more students in class B scored within 50-60 points, more students in class A scored within 90-100 points, therefore, the contrast is large. The average score of class A students is 80.125, and the average score of class B students is 71.45. The highest score for A can be as high as 98, the lowest score is 58, and the lowest score in class B is 51. It can be seen that having a high performance psychological quality and the ability to express emotions can achieve a good effect on accordion performance.

## 1. Introduction

Driven by globalization, contemporary music scholars have gradually realized that in the face of the great integration of world culture, we should not ignore the cultural characteristics of our own ethnic groups [1]. The current music education has problems such as uneven distribution of educational resources, school music courses are replaced by other majors, single curriculum teaching structure, and European music education concepts [2]. With the continuous criticism, and reference of new school intellectuals and music writers, Western music has become an irresistible social trend. Under the impact of this music trend, music education as a “victim” has unique cultural inheritance and development characteristics. The profound influence of this thought has had a direct impact on the contemporary public music aesthetics, the characteristics, content, and educational philosophy of contemporary music education. Psychology of music education is an interdisciplinary subject that has emerged in recent years. It covers the psychological knowledge of music theory, rhythm, emotion, etc., and combines the practical operation of pedagogy of subject [3]. With the reform of the education system, music teaching has gradually got rid of the predicament of being in a marginal position for a long time and has become an important part of contemporary teaching [4]. Among them, accordion performance will also be affected by it, and the performers' playing psychology and emotional expression will be affected.

RETRACTED

At first, the accordion attracted the attention of the world, and now it sings everywhere, whether it is on the stage, on the field, in the cafe, on the radio, or on the Internet, you can hear her singing [5]. The artistic significance of the accordion was recognised after the war, the great cultural revolution, reform, and opening up. The artistic level of the bass accordion has reached unparalleled heights, particularly since it was brought to our nation. International accordion art festivals, contests, performances, forums, and other events have grown in popularity in recent years, and an increasing number of students are taking home gold prizes in these competitions. The accordion business is also continually looking to diversify its development path. Many serious artists are attempting to find their unique style and have made some progress in this area [6]. The creation of the accordion's emotions during a performance is likewise an emotional art, and these feelings are inextricably linked to people's psychological processes. A process of psychological perception, comprehension, imagination, experience, and emotion goes into accordion performance [7]. Incorporating the “original work” into the individual's unique qualities is just as important as demonstrating the genuine artistic aim and passion of the piece. Each note in the dynamic secondary production is given true creative life, enhancing the musical piece and showcasing its distinct charm. Therefore, this essay suggests conducting research on how emotions are expressed through accordion playing, as well as playing psychology. The advantages of each algorithm are compared in order to provide algorithm support for accordion playing under a more objective and scientific playing psychological system, which has some reference significance for accordion playing research. The collaborative filtering algorithm and cognitive diagnosis related theories are used.

In real life, music is indispensable. People's daily life is inseparable from music, and music creation is inseparable from the emotion of life. The performance of various musical works can convey rich emotions to the audience and give the audience a good art experience feeling. Different people express their emotions in different places [8]. For example, in literature, authors express their feelings through words; in music, composers use music to express their emotions and thoughts. The accordion is a reed instrument that can perform solo and accompaniment at the same time. It can not only play single-part and multipart music but also has strong harmony [9]. Its most prominent features are rich and changeable timbre, grand sound, fixed pitch, and can interpret various types of music. Effectively conveying and expressing the emotions in accordion performance can improve the expressiveness of the tune and form a good musical image. Therefore, each accordion player must not only learn to use different playing techniques and methods but also put his own feelings into the interpretation of the works, and fully express the thoughts and emotions endowed by the original works. Infect the hearts of the audience, arouse the psychological emotional resonance of the audience, and promote the audience to enjoy the artistic enjoyment of music performance.

RETRACTED

There are various forms of emotional communication of the accordion, and performers should have a deeper understanding of it and use various performance techniques to express their emotional characteristics and emotional changes, so that they can better express their true emotions. This paper is that (1) adopts the collaborative filtering algorithm and the related theory of cognitive diagnosis and also compares the influence of the superiority of each algorithm. (2) This text research will use a variety of related algorithms to compare, so as to obtain comprehensive and in-depth research results on this topic and promote the study of the effect of accordion performance.

## 2. Related Work

The feelings of individuals can be captured and expressed through music [10]. In addition to bringing out people's joy and intoxication, music has the power to quickly awaken people to the limitless meaning of existence. People have a deep appreciation for and knowledge of music. However, as music education has been developed over time and people's cognitive abilities have increased, its worth has been increasingly recognised [11]. The same is true with playing the accordion.

Liu elaborated on the historical school education reform and its influence on music education, the important reform of school education, the historical evolution of the general school education and teaching plan, the analysis and research of teaching materials, and the appraisal of teaching materials by the Ministry of Culture. This provides a relatively broad background for the in-depth study of music education comparison [12]. Zi pointed out that the music textbook encourages and inspires people to continue to create and arrange in each of its teaching stages, so it is never finalized and ended here, but always in development, in formation, and in progress [13]. Kiilu proposed to establish a whole set of music education system, which has a wide influence in the world, and has attracted more and more attention of people in the music education circle in our country. Not only comprehensively expounds the theory and practice of the music education system but also more profoundly expounds the local development of the music education system [14]. Shubhra and Singh introduced an adaptive change factor in the teaching stage, learned from the optimal individual in the early stage, and maintained its own state better in the later stage, thereby maintaining the diversity of the population [15]. Shi and Dance's research put forward a body rhythm music teaching model that conforms to the law of development [16]. Lan conducted a systematic study on how to learn to master the classic songs of this nation [17]. Proverbio et al. pointed out that it is more important to think deeply about the substance, form, and style of the work than to practice the instrument for hours on end [18]. Erkinovna and Daughter pointed out the formation and development of cognition of musical forms, understand the expressive power of musical language and its constituent elements, and clarify the interaction and mutual connection of different artistic expression means in real music (although this mutual connection is sometimes simple, sometimes complex) and intersecting relationships, the ability to quickly grasp the characteristics of a composer's style of expression, etc., all of which are formed on the basis of experience after numerous analyses [19]. Yan believes that blindly pursuing high, difficult, and profound artistic effects in popularizing accordion education will make ordinary people intimidated, and it is difficult to achieve the original intention of popularization [20]. Shan pointed out that the various achievements in the field of accordion are a good exploration of the artistic and cultural value of the accordion, and it is the choice and direction of history, but at the same time, the popular attribute of the accordion should not be deprived, and the accordion should play a role in different cultural types and levels in the society's different roles [21].

RETRACTED

The above scholars play the accordion basically from the perspective of music itself and explore its theory and practice, influence, purpose, and music training system. They do not involve the perspective of playing psychology and rarely propose scientific education based on algorithms. Therefore, this paper will use the theory of collaborative filtering and cognitive diagnosis to study the accordion playing from the perspective of playing psychology.

## 3. Methodology

### 3.1. Basic Skills and Emotional Expression

At present, basic skills are mainly composed of basic postures and basic techniques, and basic techniques are the key to affecting the level of playing. Without basic techniques, it is impossible to express emotions.

#### 3.1.1. Basic Posture

There are two postures for playing the accordion, one is standing and the other is sitting. When playing, you should adjust the strap according to your own characteristics, so that it is in an appropriate position, it is best not to be too long, but to choose the appropriate length. Too long will make the body difficult to maintain, and will swing left and right with the pulling of the bellows when playing; if the strap is too short, the movement of the hand will be blocked when playing, which will cause tension and fatigue in the arm. The correct playing posture is beneficial to the smooth progress of playing and the catharsis of emotions.

#### 3.1.2. Basic Technology

There are three main types of accordion techniques: playing, reading music, and bellows techniques. Students must master the skills of playing and reading notation, mastering the correct keys, so they can play beautiful music as well as self-practice in accordion playing, see Figure 1. Secondly, the rational application of bellows technology. The pros and cons of using the accordion is directly related to the sound quality of the accordion. It is a medium for conveying emotions. Through different playing methods, the flowing music can be interpreted, thereby increasing the expressive power of the accordion.

There are also teaching-related factors in how well the accordion is played, as shown in Figure 2.

### 3.2. Analytical Ability and Emotional Expression

#### 3.2.1. Ability to Analyze Works

An excellent accordion player, in order to fully understand the feelings he wants to express, needs to conduct an in-depth research on its original author and creative background. For example, Mozart, Beethoven, Chopin, Mendelssohn, and other famous romantic musicians, their works are determined by their era background, social background, and life experience. Only with this quality, the player can reflect his own style in playing and perfectly display the ideas he wants to convey.

#### 3.2.2. Secondary Creative Ability

To add personal creativity to works already done by the original author is referred to as secondary creation. In order to achieve the desired effect, the performer also incorporates his or her own feelings into the performance. The performers' understanding of their works should be grounded in the context of their historical development and must not stray from their original objectives. To organically incorporate their own insights into their performances while playing, accordion musicians in the second creation must put in a lot of work, gather and improve their theoretical knowledge, and constantly widen their horizons in the middle. We can only fully express the emotion of music and play more flawless music in this way, through the second creation.

RETRACTED

### 3.3. Body Language and Emotional Expression

Body language is the extension of the performer's inner emotions to the outside, it serves the content of the performance, and body language is the most attractive one in performance activities. Therefore, the influence of an actor's body language on emotions cannot be ignored. The player's mood should change with the change of the music, and the ups and downs of the music will inevitably cause the player's mood to fluctuate, which in turn affects his body. As the rhythm of the music reaches its peak, the movements of the performer's hands and body become clearer, and the bellows become larger. If the melody of the music is gentle, the range of motion of the hands and body will be relatively low, and the opening of the bellows will also be low. Students should not only have strong arms, but also learn body language. Body language is the carrier that embodies the main thoughts and feelings of music and is an indispensable part of accordion performance, as shown in Table 1.

### 3.4. Performance Psychology and Emotional Expression

In psychology, positive psychology is a revolutionary change and a milestone in human history. And positive psychology is also widely used in the field of education along with the reform of education and teaching. Therefore, accordion music teachers in the new era must pay attention to and understand positive psychology, combine positive psychology with music teaching content, and design feasible teaching strategies, so that students can have a positive impact on music learning and keep them active in learning mentality and give full play to their advantages to create an effective music teaching, as shown in Figure 3.

Psychologists believe that negative emotions are not the same as pleasant emotions, in which they exist longer and are more complex. Positive emotions, such as happiness, can be energizing, while negative emotions, such as disgust, can lead to thoughts of vomiting; anger can lead to aggression; and fear can lead to thoughts of escape. The main connotation of positive character is character and ability, including many positive qualities. Optimists try to be more positive so that they can be happier, while negative people do the exact opposite. In order to make students form a positive personality, internal and external incentives must be organically combined, which is of great significance to teachers' education. Teachers should strengthen students' inner motivation and cultivate their inner drive. When students have a strong interest in what they are learning, their learning purpose will turn to intellectual curiosity, so that they will generate positive motivation, such as intellectual curiosity, enthusiasm, and perseverance.

RETRACTED

Every accordion player experiences a variety of psychological changes in perception, memory, emotion, rationality, imagination, intuition, and more when they play.

#### 3.4.1. On-the-Spot Performance Psychology

Each live performance is a unique, exclusive, repeating performance that calls for actors to have a positive outlook and the capacity to adapt to changes. Anyone who plays the accordion will feel neurotic before beginning, especially in the beginning. The performance will lose its initial level under conditions of extreme anxiety, and it may even be halted by deviations or mistakes. Along with continuously honing one's own playing abilities, one must also constantly train their “normal heart” in order to overcome the issues that arise during live performances. Daily practice is vital to the emotion that a player displays when playing. It is impossible to play on stage as a performer. Long hours of practice, ongoing research, analysis, and application are required. When playing on stage, an accomplished accordion player must feel comfortable. He is only able to manage the game's rhythm while playing. He can readily repair his faults while playing, which allows him to both play while feeling the audience's emotions and to experience his own a good job at expressing their feelings.

#### 3.4.2. Confidence in Playing Psychology

Meitner also reminded his colleagues to be confident in their choice of subject matter. From Meitner's practice, we can see that in the process of artistic creation, self-confidence is essential. When creating art, you must have confidence in your own thoughts, your own choices, and your own judgments. In a sense, believing your thoughts and affirming your actions is a great way to motivate your inner autosuggestion, and it has a big impact on the nature of your creative actions and the final outcome. Self-confidence is a basic quality that everyone must have when doing anything, so when playing, performers need to be confident when they play and show their best to the audience. So, give yourself a boost before you play, then let go of the distractions while you play, stay confident, and be confident that you are playing the best. In daily training, we should strengthen the exercise in this are and always believe in ourselves and have confidence.

RETRACTED

#### 3.4.3. Focus on Playing Psychology

We all know that when a person is fully concentrated, he will integrate his attention, knowledge of the work, and knowledge of the work into the work. In the process of playing, he will always maintain confidence, integrate your soul into the music, integrate with the music, and let your state achieve the best effect. As the modern Russian violinist and conductor Spivakov said “an actor should know very clearly what he is going to do on stage, and try to make himself understand his creative mission and goal”. In the process of artistic creation, we should focus all our attention on the goals and objectives of creation, and the accordion player should concentrate on playing, expressing his emotions perfectly, and letting his body fully immerse himself in the music to get the best results from his playing.

### 3.5. Collaborative Filtering Algorithm

The core of the collaborative screening algorithm is collaboration, that is, to provide similar samples to the target samples. Collaborative filtering algorithms mainly include user collaboration and project collaboration. For example, according to the collaborative screening of products, since the user's evaluation of the product is a sparse matrix, the evaluation of the product by many users is unclear. Therefore, we need to determine whether the user has evaluated a certain item, that is, the item's rating and the similarity between that item. Finding similarities in similar samples is called collaborative screening. On the basis of the traditional cooperative filtering algorithm, an algorithm based on machine learning and a CNN algorithm based on deep learning are proposed. This section will detail two common collaborative filtering algorithms.

According to the collaborative filtering algorithm of the target user, according to the user's preference, users who use the same item must have the same preference, so the same item can be recommended to the user. For example, users can be matched according to their favorite music mechanism.

Accordion playing form for each student before recommending an accordion playing form, the system first finds a set of other students with similar interests to the target student. The following formula can be used to calculate the similarity of students' interests.

(1) $$\begin{array}{c} S_{\text{ab}}=\left\{N\left(a\right)\text{nN}\left(b\right)\right\}. \end{array}$$

In the formula, the *S*_ab_ representative of *a* and *b* is the similarity of two students and *N*(*a*) and the set of *N*(*b*) are the accordion playing forms that student *a* and student *b* have had positive feedback, respectively.

RETRACTED

After obtaining the similarity of students' interests, the following formula can be used to calculate the students' interest in a certain form of accordion performance.

(2) $$\begin{array}{c} X\left(a,i\right)=\underset{\text{beS}\left(a,m\right)\text{nN}\left(i\right)}{\left\{S_{\text{ab}}\;R_{\text{bi}}\right\}}. \end{array}$$

The formula *X*(*a*, *i*) expresses the students' interest in the *a* form of playing *i* the accordion, *S*(*a*, *m*) including students who are *a* close to the students' interests, is the *N*(*i*) set of student users who have acted on the *S*_ab_ form of resources, and *i* is the similarity of interests between *R*_bi_ student *a* and student *b*, which means the student *b*'s interest in the form of resources *i* spend.

Using the above method, the system can understand the students' interest in a certain form of accordion playing. The system can then try to recommend an appropriate accordion playing form for the student and package the knowledge content through this accordion playing form.

Accordion performance teaching adopts the method of item-based collaborative filtering and selects and recommends pertinent accordio-packed performance topics for each student. These selected performance topics can help students to quickly improve their performance skills. Throughout the course, many topics are related to a certain extent. The correlation between performance topics can be calculated by the following formula:

(3) $$\begin{array}{c} Q_{\text{uv}}=\left|F\left(u\right)\text{nF}\left(v\right)\right|,\\ T_{\text{au}}=V^{\left|F\left(u\right)\right|\left|F\left(v\right)\right|}. \end{array}$$

In the formula, the *Q*_*uv*_ representative of *u* and *v* is the correlation between the |*F*(*u*)*nF*(*v*)| two subjects which represent the number of *v* students who performed poorly at the *u* same time. After obtaining the similarity of the subject, the error rate parameter *a* of the student's performance *v* can be predicted by the calculation formula shown below.

(4) $$\begin{array}{c} Y\left(a,v\right)=\underset{\text{ueF}\left(u\right)\text{nQ}\left(y,K\right)}{\left\{Q_{\text{uv}}\;T_{\text{au}}\right\}}. \end{array}$$

In the formula, *Q*(*a*, *v*) is the set *Q*_uv_ of topics *V* with the *v* highest degree of relevance to *K* the subject, *u* is the degree of relevance between the subject and the subject, and *T*_au_ is the *u* of the student *a*'s error rate parameter for the subject.

RETRACTED

Using the above method, the system can understand the importance of a topic to a student. The system can then try to recommend targeted topics for that student. Of course, in order to avoid lowering students' self-confidence, the system can also appropriately provide some topics that students can easily play better.

German psychologists found that forgetting begins immediately after a performance, and the forgetting process is not uniform. The speed of forgetting is fast at first, and then gradually slows down.

The input information becomes the short-term memory of people after learning through the process of human attention, but if it is not played in time, these memorized things will be forgotten, and after a timely performance, these short-term memories will be forgotten. The memory of time will become a kind of long-term memory of a person, as shown in Figure 4.

Additionally, it is thought that every pupil should have a unique memory in this setting. Each performance should have an impact based on the student's memory, how many times he has played, how much time has passed between the two performances, and how challenging the knowledge point was. Since student memory is hard to quantify mathematically, IQ scores, historical average grades, and online learning activities—in which IQ scores are determined through online question-and-answer tests—are used in its stead. The number of days a pupil can retain a memory after each performance can be determined using the formula below.

(5) $$\begin{array}{c} T=aM^{2}+bN^{2}+cO^{2}+dP^{2}+eQ^{2}+fR^{2}. \end{array}$$

In the above formula, *T* represents the number of days to keep memory. After *T* days have passed, the system will arrange the students for the next performance. *M* indicates the number *N* of times played: indicates the time interval between this *O* performance and the last performance; indicates the student's IQ value; *P* indicates the student's average score in the past; *Q* indicates the student's online learning activity; and *R* indicates the difficulty level of the knowledge point. *a*, *b*, *c*, *d*, *e*, and *f* are the weights of each parameter, and their initial values can be set to 2, 1.5, 0.05, 0.05, 0.05, and 0.05, respectively. These weights can be continuously revised through the analysis of campus big data.

At each performance, the system will quiz the students and adjust the weights according to the quiz results. If the student's performance is satisfactory, the network uses the following formula as the objective function. Where the initial value of *p* is 0.2,

(6) $$\begin{array}{c} E_{d}={\left(p+2\right)}^{2}. \end{array}$$

If the student's performance is not good, the network adopts the following formula as the objective function. Where the min function obtains the minimum value,

(7) $$\begin{array}{c} E_{d}=-\min\left(T-{\left(pT+2\right)}^{2}\right). \end{array}$$

RETRACTED

### 3.6. Theories Related to Cognitive Diagnosis

In recent decades, the rapid development of educational data mining (EDM) has promoted the advancement of teaching resource recommendation. The purpose of EDM is to automatically extract information from a large amount of data information generated or related to people's learning behaviors in educational and teaching environments. Valuable information and teaching resource recommendation is to combine data mining, artificial intelligence, Internet, recommendation system, and other technologies to actively recommend these valuable information to users according to the individual needs of learners.

Cognitive diagnosis is a modern educational psychometric theory formed by combining educational psychometric and cognitive psychology. It is based on the Q matrix of cognitive characteristics and aims to describe subjects by discovering their (usually student users) underlying knowledge status and levels of cognitive abilities such as a skill. Cognitive diagnosis is a science based on modern computer technology and statistical analysis, which can diagnose the cognitive structure and behavior of subjects. At present, in the actual education and teaching practice, people generally adopt the method of cognitive diagnosis, which makes the traditional online classroom teaching develop towards a more personalized direction. According to incomplete statistics, there are currently more than 80 related cognitive diagnostic models. Some models assume the continuity of attributes, and some models assume the discreteness of attributes. Among them, the most commonly used are Item Response Theory (IRT) and potential classification.

Item Response Theory (IRT) is used to describe the relationship between subjects' abilities and item characteristics. It breaks through the limitations of traditional classical measurement theories and is a new and modern educational psychometric theory. Item Response Theory will test users. The potential cognitive ability level (such as student users) is parameterized and modeled by combining the user's behavioral performance on test items (such as test questions, knowledge points, and learning videos.). The item response theory model holds that there is a functional relationship between students' cognitive ability level and their performance in teaching resources and is defined as item response function. The basic models of item response theory mainly include one-parameter, two-parameter, and three-parameter logistic models, as shown in the following formulas, respectively, and in Table 2.

(8) $$\begin{array}{c} P\left(u_{\text{ij}}=1\left|\theta_{i}\right.\right)=\frac{e^{\left(\theta_{i}-d_{j}\right)}}{1+e^{\left(\theta_{i}-d_{j}\right)}},\\ P\left(u_{\text{ij}}=1\left|\theta_{i}\right.\right)=\frac{1}{1+e^{-da_{j}\theta_{i}-d_{j}}},\\ P\left(u_{\text{ij}}=1\left|\theta_{i}\right.\right)=g_{j}+\frac{1-g_{j}}{1+e^{-Ca_{j}\left(\theta_{i}-d_{j}\right)}}. \end{array}$$

Generally speaking, assuming that the current project parameters are known to perform the maximum likelihood estimation of the capability parameters, or assuming that the current capability parameters are known to perform the maximum likelihood estimation of the project parameters, use the maximum likelihood to estimate the capability parameters of the IRT model and the project parameters. The alternating estimation approach is used to estimate the IRT model parameters when both the capability parameters and the project parameters are unknown. These are the general steps:

1. Obtain the score matrix of the tested users and items
2. Parameter estimation

If the difficulty coefficient, guessing coefficient, and discrimination coefficient of the current item are all known, the answer result data in the score matrix and the known difficulty coefficient, guessing coefficient, and discrimination coefficient are substituted into the IRT model, and the maximum likelihood function of the ability parameter is established, as indicated by

(9) $$\begin{array}{c} L=\overset{m}{\underset{i=1}{\prod }}p_{i}^{y_{i}}{\left(1-p_{i}\right)}^{1-y_{i}}. \end{array}$$

Among them is the correct answer probability obtained by the IRT model function, which is the real answer situation of the tested user in the score matrix. Taking the logarithm of both sides, we get

(10) $$\begin{array}{c} \ln\left(L\right)=\overset{m}{\underset{i=1}{\sum }}y_{i}\ln\left(p_{i}\right)+\left(1-y_{i}\right)\ln\left(1-p_{i}\right). \end{array}$$

One of the most often employed models for cognitive diagnostics is the deterministic input and noise gate model (DINA), which is a typical representative model in latent classification models. A straightforward random connection model is the DINA model. The model only has two parameters, the error factor and the guess factor, compared to previous models. It is more adaptable, succinct, and simple to understand when compared to other models. As a result, it has been extensively used and researched by experts in the field. Formula is the mathematical representation of the DINA model

(11) $$\begin{array}{c} P\left(u_{ij}=1\left|\alpha_{i}\right.\right)={\left(1-s_{j}\right)}^{\xi_{ij}}{g_{j}}^{1-\xi_{ij}}. \end{array}$$

The left side of Formula (11) *P*(*u*_*ij*_ = 1|*α*_*i*_) is the probability that *g*_*j*_ = *P*(*u*_*ij*_ = 1|*ξ*_*ij*_ = 0) the subject can correctly answer the item with the *j* accordion playing mastery level. *α*_*i*_ indicates the guessing probability of a student *i*'s good performance, that is, the probability that a student can perform well when he does not fully grasp all the knowledge points and abilities examined in the performance *j*. *s*_*j*_ = *P*(*u*_*ij*_ = 0|*ξ*_*ij*_ = 1) represents the probability of mistakes in the performance of students, that is, the probability of wrong performance when students *i* have mastered all the knowledge points and abilities examined in performance *j*. Among them, *ξ*_*ij*_ the mathematical expression *ξ*_*ij*_ that indicates whether students *i* fully master all the knowledge points (attributes) and abilities of the performance investigation is shown *j* in

(12) $$\begin{array}{c} \xi_{\text{ij}}=\overset{l}{\underset{k=1}{\prod }}\alpha_{\text{ik}}^{q_{\text{jk}}}. \end{array}$$

Among them, it means *ξ*_ij_ = 1 that the tested user (student user) has *i* mastered all the knowledge points and abilities (skill attributes) examined by accordion playing *j*, on the contrary, *ξ*_ij_ = 0 means that the tested user (student user) has *i* not fully mastered all the knowledge points and abilities examined by the accordion (attribute skill).

RETRACTED

## 4. Results Analysis and Discussion

In the experiment method, this study chooses 70%, 50%, 30%, and 10% of all data sets as test data sets, while the remaining data sets are used as training data sets to observe different data sparse degrees of applying different algorithms and evaluate their impacts. To put it another way, if 70% of the data is randomly chosen as the test data, then the remaining 30% is used as the training set to anticipate the test set data, and the same is true for 50%, 30%, and 10%. The accordion performance resources are also classified into simple and compound performance resources within the range of the difficulty value of 0.6, and a comparison study of the recommendations effects of various difficulty performance resources is conducted. While some video performance resources and text performance resources are carefully annotated by subject-matter experts or teachers who produce the resources, other student historical response materials are video performance resources.

Figures 5 and 6 show that the CUPMF model consistently outperforms the other four algorithms in terms of the accuracy of recommendations for simple performance resources and complex performance resources as the test set ratio is continuously decreased, i.e., as the training set ratio is continuously increased. The F1 value is specifically 8.6% higher when proposing simple performance resources than the other four algorithms as a whole, and it can reach 0.888 when the test set is 10%. The F1 value is also higher while recommending complex performance resources than the other four algorithms. An increase of 5.6% on average, reaching 0.958 when the test set is 10%. The aforementioned findings demonstrate how well the CUPMF algorithm works to increase recommendation outcomes and suggestion accuracy. Among them, the CUPMF model is based on a joint probability model, combining deep learning technology and algorithms, which can guarantee a high recommendation accuracy even when the number of student users is sparse. Additionally, the CUPMF model is based on a joint probability model, combining deep learning technology and algorithms, which results in higher diagnostic accuracy.

RETRACTED

From the above chart, the superiority of each algorithm can be compared, and the superiority of the CUPMF algorithm in accordion performance is obtained in this paper. The test results of the five algorithms are statistically tested, and the final superiority results are shown in Figure 7. Statistical tests show that CUPMF ranks first in the superiority test. There are significant differences between the solutions obtained by the five algorithms of CUPMF, RBF, GWO, MA, and MFO and the known optimal values, while the difference between the results of CUPMF and the known optimal results is the smallest, which intuitively shows that CUPMF It is better than the five algorithms of RBF, GWO, MA, and MFO, and gives the best results known so far.

The following is an example analysis of accordion performance based on playing psychology and emotional expression. The research group has set up group B (unstable psychological impact) and group A (stable psychological impact). The study group organized students into two groups I and II: there were 717 students in group I and 734 students in group II. 36 students were randomly selected to test the performance of groups A and B.

As can be seen from Figure 8, the overall trend of the average performance of the students in group A and group B is similar, both within 50-100 points. However, there is still a certain difference in the performance scores of the two groups of students. Most of the accordion scores of the students in group A were higher than those of the students in group B, up to 36 points higher, and most of them were higher than 10 points. But group B students also have higher performance scores. Due to the randomness of randomly selected students, they will be divided into A and B classes for a comprehensive investigation (emotional expression and performance psychology).

RETRACTED

As can be seen from Figure 9, the overall trend of the average performance of the accordion students in the two classes is quite different. The performance of the students in class A is obviously better than that of the students in class B. Of course, there are some students in class B who are more outstanding. However, there are more students in class B who are within 50-60 points, while students in class A have more students who are within 90-100 points, the contrast is large. The average score of class A students is 80.125, and the average score of class B students is 71.45. The highest score for A can be as high as 98, the lowest score is 58, and the lowest score in class B is 51. It can be seen that having a high performance psychological quality and the ability to express emotions can achieve a good effect on accordion performance.

## 5. Conclusion

Overall, sound accordion playing technique is essential to the performance process, but playing technique alone is insufficient. Starting with performing abilities, we must further comprehend the connotation of music, analyse it from the perspectives of theory, inventive personality, music language, music psychology, etc., before music can properly communicate the feelings we wish to express to interpret music, one's own creative literacy. The expression of emotion is the essence of performing arts, and without it, a performance cannot touch the hearts of the audience. In order to increase your artistic quality overall and create the ideal state of music, you must carefully comprehend each play's meaning as well as the thoughts and emotions it seeks to convey. The performance of the performance is greatly influenced by the accordion player's mental condition. Formally speaking, a person's psychological quality is both innate and acquired when they play the accordion. We must develop a positive attitude in our everyday training, modify our psychological pressure, and make sure that we keep that positive attitude throughout the performance.

### 5.1. Self-Regulation before Live Performance

Before the live performance, in the usual training, you should focus on cultivating your self-confidence. Sometimes, tension is caused by lack of self-confidence and strong desire to perform, which leads to anxiety. Therefore, when exercising, pay more attention to your strengths to enhance your confidence. At the same time, it is necessary to combine effective memory technology with music memory, organically combine the three memories of sports, video, hearing, and intelligence, and firmly remember the music; secondly, the venue, equipment, clothing, and hairstyle must be prepared in advance., Actors want to perform on the stage, they must be familiar with the lighting, sound and control system of the stage in advance to achieve the effect of improvisation.

RETRACTED

### 5.2. Psychological Regulation during Live Performance

First, when you play, try to concentrate as much as possible. Do not be swayed by the audience, whether it is sound or action, be completely immersed in the music. Do not think about how to overcome technical difficulties and do not think about how to make the audience accept your performance, let alone if you do not perform well, or if the audience does not like you. The moment he played the first note, he was immersed in the piece. At the same time, the atmospheric stage manners and body movements will also unconsciously improve the performers' self-confidence and reduce physical and mental pressure. Finally, to have a sense of excitement, most actors will show some excitement and nervousness before the performance. We need to convert these pressures and excitements into performance motivation, and let the music express naturally in our hearts, so as to achieve good performance results.

### 5.3. Post-Performance Feedback and Reflection

The summary and thinking after the performance is often overlooked by the actors. Whenever we finish playing, we must analyze and summarize to the teachers and classmates. If you can play it, you should sum up your experience so that you can perform better and better next time. If it is a failed performance, you should analyze your mistakes more, find out the reasons, reduce your psychological pressure and reduce your tension, so that you can achieve a breakthrough in the next performance. Whether it is success or failure, he must stand on an objective stand so that he can better understand his performance.

## Figures and Tables

**Figure 1:** Factors such as self-practice in accordion performance.

**Figure 2:** Factors influencing accordion teaching.

**Figure 3:** Psychology-music classroom construction.

**Figure 4:** Learning structure neural network.

**Figure 5:** F1 value table of simple performance resource prediction results.

**Figure 6:** F1 value table of complex performance resource prediction results.

**Figure 7:** Advantages of each algorithm.

**Figure 8:** Comparison of the performance effects of group A and group B.

**Figure 9:** The comprehensive scores of accordion performances of class A and class B.

**Table 1:** Comparison of the accordion with other instruments.

Musical instrument	Difficulty
Accordion	The hardest (the most stamina)
Other musical instruments	Including easy, normal, and difficult

RETRACTED

**Table 2:** IRT model formula parameter correspondence table.

Parameter	Definition	Brief introduction
*a*_*j*_	Test item discrimination coefficient	Indicates the degree of discrimination of test items or questions and determines the slope of the middle of the curve in the curve. The smaller the value is, the harder it is to distinguish the test scores of the tested users.
*d*_*j*_	Difficulty factor of test items	Indicates the difficulty of the tested item or question, and the displacement in the direction of the horizontal axis of the curve is represented in the curve. The greater the difficulty coefficient, the higher the ability is required for the subject to obtain a higher score.
*g*_*j*_	Test item guess factor	Indicates the probability that the tested user will answer the test question without prior knowledge of the test item, such as a multiple-choice question with a certain probability of being right.
*θ*_*i*_	The potential ability value of the testee	Indicates the subject's mastery of the knowledge points or abilities to be assessed by the project or topic.
*C*	Constant 1.702	Ordinary constants.

## Data Availability

The data used to support the findings of this study are available from the corresponding author upon request.
